This article has been retracted.

# Long noncoding RNA *VPS9D1-AS1* augments the malignant phenotype of non-small cell lung cancer by sponging microRNA-532-3p and thereby enhancing *HMGA2* expression

**DOI:** 10.18632/aging.102628

**Published:** 2020-01-05

**Authors:** Xiao Han, Tianren Huang, Junqing Han

**Affiliations:** 1 Guangxi Medical University, Cancer Hospital, Nanning 530021, China; 2 Cancer Center, Shandong Provincial Hospital Affiliated to Shandong University, Jinan 250021, China

**Keywords:** non-small cell lung cancer, microRNA-532-3p, high mobility group AT-hook 2, *VPS9D1-AS1*

## Abstract

We investigated the influence of the long noncoding RNA VPS9D1 antisense RNA 1 (*VPS9D1-AS1*) on the malignant phenotype of non-small cell lung cancer (NSCLC) cells *in vitro* and *in vivo*. We also explored the mechanisms by which *VPS9D1-AS1* exerts its oncogenic action during NSCLC progression. *VPS9D1-AS1* expression was upregulated in NSCLC; the extent of its upregulation significantly correlated with patients’ adverse clinicopathological characteristics and shorter overall survival. When *VPS9D1-AS1* was knocked down in NSCLC cells, their proliferation, colony-forming capacity, migration, and invasiveness were lower, whereas their apoptosis rate was higher, compared to the control. *VPS9D1-AS1* knockdown attenuated tumor growth of NSCLC cells *in vivo*. Mechanistically, *VPS9D1-AS1* directly interacted with microRNA-532-3p (miR-532-3p) in NSCLC cells; the impact of *VPS9D1-AS1* knockdown on NSCLC cells was attenuated by miR-532-3p inhibition. Furthermore, *VPS9D1-AS1* knockdown decreased the expression of high mobility group AT-hook 2 (*HMGA2*) in NSCLC cells via miR-532-3p sponging. Recovery of *HMGA2* expression partially reversed the inhibitory effects of *VPS9D1-AS1* knockdown on NSCLC cells. Thus, *VPS9D1-AS1* functions as a competing endogenous RNA that positively regulates *HMGA2* expression by sponging miR-532-3p in NSCLC cells, suggesting that the *VPS9D1-AS1*–miR-532-3p–*HMGA2* pathway can be a potential diagnostic and/or therapeutic target in NSCLC.

## INTRODUCTION

Lung cancer is the third most prevalent type of human malignant tumor and a leading cause of cancer-related death among both men and women globally (~18%) [1]. It was estimated that lung cancer was responsible for approximately 2.1 million new cancer cases and 1.8 million deaths worldwide in 2018 [2]. Lung cancer is classified into two types: small cell lung cancer and non-small cell lung cancer (NSCLC) [3]. NSCLC, which accounts for approximately 85% of all lung cancer cases, includes three subtypes, namely adenocarcinoma, squamous cell carcinoma, and large cell carcinoma [4]. Over the past several decades, there have been tremendous advances in targeted therapeutic techniques and the development of new anticancer compounds; however, NSCLC is still one of the most frequent and deadly malignant tumors with a 5-year overall survival rate below 18% [5]. Uncontrolled growth, local/distant metastasis, and recurrence are responsible for the unsatisfactory clinical outcomes of patients with NSCLC [6]. Hence, a more comprehensive understanding of NSCLC pathogenesis is of paramount importance for the identification of novel promising therapeutic targets in this disease.

Long noncoding RNAs (lncRNAs) represent a family of RNAs that are over 200 nucleotides long but have no protein-coding ability [7]. LncRNAs function as guides, scaffolds, and molecular sponges in their interactions with proteins, microRNAs (miRNAs), and mRNAs, thereby creating complex networks that regulate various physiological and pathological processes, including cancer initiation and progression [8]. Recently, several studies revealed the contribution of lncRNAs to the formation and progression of multiple types of cancers, including NSCLC [9–11]. A large number of lncRNAs are expressed abnormally in NSCLC, e.g., *HOXA-AS2* [12], *LEF1-AS1* [13], and *BLACAT1* [14]. LncRNAs exert either antitumor or tumor-promoting actions in NSCLC and modulate various pathological and physiological processes, including cell proliferation, cell cycle, apoptosis, metastasis, angiogenesis, and epithelial–mesenchymal transition [15, 16].

miRNAs are another group of noncoding RNA molecules; they are RNAs that are 17–24 nucleotides long [17]. They modulate gene expression via direct interaction with the 3′-untranslated region (3′-UTR) of their target mRNAs, thus leading to either mRNA degradation or translational inhibition [18]. Over 2,000 miRNA genes have been identified in the human genome; these miRNAs are estimated to regulate approximately 30% of all protein-coding genes [19]. Aberrations in the expression of miRNAs involved in tumor-suppressive or oncogenic processes have been widely reported in NSCLC [20–22]. Therapies that target lncRNAs and/or miRNAs may be potentially used for effective NSCLC management.

Changes in the expression of the lncRNA *VPS9D1-AS1* have been observed in several malignant tumors, including gastric [23], prostate [24], and colorectal [25] cancers. Expression of *VPS9D1-AS1* is upregulated in NSCLC and closely associated with clinical outcome [26]. Nevertheless, the manner in which *VPS9D1-AS1* regulates NSCLC progression and the mechanisms of its action remain poorly understood. Hence, the present study was designed to investigate the relationship between the expression level of *VPS9D1-AS1* and the malignant characteristics of NSCLC cells both *in vitro* and *in vivo*. In addition, the mechanisms by which *VPS9D1-AS1* exerts its oncogenic effects during NSCLC progression were explored.

## RESULTS

### High level of *VPS9D1-AS1* expression in NSCLC

Expression profiles of *VPS9D1-AS1* in 51 pairs of NSCLC samples and corresponding normal lung tissues were evaluated using reverse transcription-quantitative polymerase chain reaction (RT-qPCR). *VPS9D1-AS1* expression was higher in NSCLC tissue samples than in normal lung tissues (Figure 1A, *P* < 0.05). By using the median level of *VPS9D1-AS1* expression in the NSCLC tissue samples as a cutoff, all samples from the 51 NSCLC patients were classified into either *VPS9D1-AS1* high-expression or *VPS9D1-AS1* low-expression groups. The analysis of the correlation between *VPS9D1-AS1* expression level and clinicopathological characteristics revealed that increased *VPS9D1-AS1* expression correlated significantly with tumor size (*P* = 0.025), TNM stage (*P* = 0.002), and lymph node metastasis (*P* = 0.012; Table 1). In particular, patients with NSCLC in the *VPS9D1-AS1* high-expression group showed shorter overall survival than patients in the *VPS9D1-AS1* low-expression group (Figure 1B, *P* = 0.030). Furthermore, the expression of *VPS9D1-AS1* was measured using RT-qPCR in five NSCLC cell lines (H522, H460, H1299, A549, and SK-MES-1). The normal, non-tumorigenic, bronchial epithelium cell line BEAS-2B was chosen as the control. *VPS9D1-AS1* expression levels were higher in all tested NSCLC cell lines than in BEAS-2B cells (Figure 1C, *P* < 0.05). These data indicated that *VPS9D1-AS1* is upregulated in NSCLC and that its expression level may correlate with tumor progression.

**Figure 1:** **High expression of *VPS9D1-AS1* in NSCLC indicating poor prognosis in NSCLC patients.** (**A**) RT-qPCR analysis of *VPS9D1-AS1* expression in 51 pairs of NSCLC samples and corresponding normal lung tissues. *P < 0.05 vs. normal lung tissues. (**B**) Relationship between *VPS9D1-AS1* expression and overall survival of patients with NSCLC analyzed by the Kaplan–Meier method and log-rank test. *P* = 0.030. (**C**) Determination of *VPS9D1-AS1* expression by RT-qPCR in total RNA from five NSCLC cell lines (H522, H460, H1299, A549, and SK-MES-1) and one normal nontumorigenic bronchial epithelium cell line (BEAS-2B). *P < 0.05 vs. BEAS-2B cells.

**Table 1:** Correlation between *VPS9D1-AS1* expression and clinicopathological characteristics of patients with non-small cell lung cancer.

**Clinicopathological characteristics**	***VPS9D1-AS1* expression**		***P*-value**
	**High (*n* = 26)**	**Low (*n* = 25)**	
**Gender**			0.164
Male	15	9	
Female	11	16	
**Age (years)**			0.779
<60	12	10	
≥60	14	15	
**Smoking history**			0.267
Smokers	16	11	
Never smokers	10	14	
**Tumor size (cm)**			0.025
<3	7	15	
≥3	19	10	
**TNM stage**			0.002
I–II	6	17	
III–IV	20	8	
**Lymph node metastasis**			0.012
Negative	9	18	
Positive	17	7	

### *VPS9D1-AS1* knockdown inhibits the proliferation, migration, and invasiveness of NSCLC cells and promotes their apoptosis

The observed relationship between *VPS9D1-AS1* expression level and malignancy prompted us to investigate the biological effects of *VPS9D1-AS1* on the malignant phenotype of NSCLC H460 and A549 cells, which showed the highest expression of *VPS9D1-AS1* among the five NSCLC cell lines. H460 and A549 cells were transfected with the small interfering RNA (siRNA) *si-VPS9D1-AS1* targeting *VPS9D1-AS1* or negative control siRNA (si-NC). Successful knock-down of *VPS9D1-AS1* after transfecting H460 and A549 cells with *si-VPS9D1-AS1* was confirmed by RT-qPCR (Figure 2A, *P* < 0.05).

**Figure 2:** ***VPS9D1-AS1* knockdown inhibits proliferation, colony-forming capacity, migration, and invasiveness of H460 and A549 cells but promotes their apoptosis**. (**A**) Evaluation of the transfection efficiency of H460 and A549 cells with *si-VPS9D1-AS1* or si-NC at ~48 h post-transfection using RT-qPCR. *P < 0.05 vs. the si-NC group. (**B**–**D**) Differences in the proliferation, colony-forming capacity, and apoptosis rate of H460 and A549 cells transfected with *si-VPS9D1-AS1* or si-NC determined by the CCK-8 assay, the colony formation assay, and flow cytometry, respectively. *P < 0.05 vs. the si-NC group. (**E**, **F**) Effects of treatment with *si-VPS9D1-AS1* or si-NC on the migration and invasiveness of H460 and A549 cells assessed by the Transwell migration and invasiveness assays, respectively. *P < 0.05 vs. the si-NC group.

Cell Counting Kit-8 (CCK-8) and colony formation assays showed that the proliferative (Figure 2B, *P* < 0.05) and colony-forming (Figure 2C, *P* < 0.05) capabilities of both H460 and A549 cells were significantly attenuated by *VPS9D1-AS1* knockdown. Flow cytometry revealed that H460 and A549 cells transfected with *si-VPS9D1-AS1* manifested a higher rate of apoptosis than those transfected with si-NC (Figure 2D, *P* < 0.05). These data suggested that the decrease in NSCLC cell proliferation induced by *VPS9D1-AS1* knockdown was due to apoptosis induction. Transwell migration and invasiveness assays showed that transfection with *si-VPS9D1-AS1* significantly decreased the migratory (Figure 2E, *P* < 0.05) and invasive (Figure 2F, *P* < 0.05) capabilities of H460 and A549 cells. Overall, these results suggested that *VPS9D1-AS1* expression may exert oncogenic effects in NSCLC cells *in vitro*.

### *VPS9D1-AS1* acts as a molecular sponge of miR-532-3p in NSCLC cells

Numerous cytoplasmic lncRNAs can function as competing endogenous RNAs (ceRNAs) by competitively binding to specific miRNAs [27]. To elucidate the molecular mechanisms underlying the oncogenic effects of *VPS9D1-AS1* in NSCLC cells, we first investigated the subcellular localization of *VPS9D1-AS1* in NSCLC cells. *VPS9D1-AS1* was mainly localized in the cytoplasm of H460 and A549 cells (Figure 3A, *P* < 0.05), suggesting that this lncRNA may function as a ceRNA of some miRNAs in NSCLC. To test this hypothesis, potential interactions between *VPS9D1-AS1* and miRNAs were explored using bioinformatics analysis. We focused on the changes in the expression of miR-532-3p as our analysis predicted that this miRNA (Figure 3B) has a high probability of binding to *VPS9D1-AS1*; in addition, miR-532-3p has been reported to play a crucial role in NSCLC progression [28].

**Figure 3:** ***VPS9D1-AS1* functions as a sponge for miR-532-3p in NSCLC cells.** (**A**) Relative expression of *VPS9D1-AS1* in nuclear and cytoplasmic fractions of H460 and A549 cells determined by subcellular fractionation and RT-qPCR analysis. (**B**) Predicted wild-type and mutant complementary sites of miR-532-3p in a *VPS9D1-AS1* fragment. (**C**) RT-qPCR analysis of miR-532-3p expression in 51 pairs of NSCLC samples and corresponding normal lung tissues. *P < 0.05 vs. normal lung tissues. (**D**) Negative correlation between *VPS9D1-AS1* and miR-532-3p levels in the 51 NSCLC tissue samples revealed by the Spearman’s rank correlation analysis. R^2^ = 0.3370, *P* < 0.0001. (**E**) RT-qPCR analysis of miR-532-3p expression levels in H460 and A549 cells with *VPS9D1-AS1* knockdown. *P < 0.05 vs. the si-NC group. (**F**) RT-qPCR analysis of miR-532-3p expression levels in H460 and A549 cells transfected with agomir-532-3p or agomir-NC. *P < 0.05 vs. the agomir-NC group. (**G**) Interaction between miR-532-3p and VPS9D1-AS1 in NSCLC cells revealed by the luciferase reporter assay. H460 and A549 cells were co-transfected with a luciferase reporter plasmid carrying wild-type (wt) or mutant (mt) VPS9D1-AS1 and agomir-532-3p or agomir-NC. *P < 0.05 vs. the agomir-NC group. (**H**) miR-532-3p and VPS9D1-AS1 enrichment in AGO2 immunoprecipitates from H460 and A549 cell lysates determined by the RIP assay. IgG served as negative control. *P < 0.05 vs. the IgG group.

To examine the correlation between *VPS9D1-AS1* and miR-532-3p expression levels in NSCLC, miR-532-3p expression levels were quantified by RT-qPCR in 51 pairs of NSCLC samples and corresponding normal lung tissues. We found that miR-532-3p expression was lower in NSCLC tissue samples than in normal lung tissue samples (Figure 3C, *P* < 0.05). Of note, an inverse correlation between *VPS9D1-AS1* and miR-532-3p expression levels was observed in NSCLC tissue samples, as evidenced by Spearman’s rank correlation analysis (Figure 3D; R^2^ = 0.3370, *P* < 0.0001). We also examined whether miR-532-3p expression was affected by *VPS9D1-AS1* levels in NSCLC cells and established that *VPS9D1-AS1* knockdown significantly increased miR-532-3p expression in H460 and A549 cells (Figure 3E, *P* < 0.05).

Direct binding of miR-532-3p to *VPS9D1-AS1* in NSCLC cells was verified by the luciferase reporter assay. Luciferase reporter plasmids carrying the wild-type (wt) or mutant (mut) binding site for miR-532-3p were constructed (VPS9D1-AS1-wt and VPS9D1-AS1-mut, respectively) and separately co-transfected with agomir-532-3p, an miR-532-3p mimic increasing its expression, or agomir-NC into H460 and A549 cells. Agomir-532-3p transfection-mediated upregulation of miR-532-3p (Figure 3F, *P* < 0.05) dramatically decreased VPS9D1-AS1-wt luciferase activity (*P* < 0.05) in H460 and A549 cells, whereas no such change was detected in cells transfected with VPS9D1-AS1-mut (Figure 3G). An RNA immunoprecipitation (RIP) assay confirmed that *VPS9D1-AS1* and miR-532-3p were substantially enriched in the immunoprecipitated AGO2 protein complex, suggesting that AGO2 bound to *VPS9D1-AS1* and miR-532-3p directly in NSCLC cells (Figure 3H, *P* < 0.05). Collectively, these data provided sufficient evidence that *VPS9D1-AS1* directly interacts with miR-532-3p in NSCLC cells.

### *HMGA2* is a direct target gene of miR-532-3p in NSCLC cells

To explore the biological effects of miR-532-3p on NSCLC tumorigenesis, agomir-532-3p or agomir-NC was introduced into H460 and A549 cells. Next, the influence of miR-532-3p upregulation on cell proliferation was examined using the CCK-8 and colony formation assays. Ectopic miR-532-3p expression strongly decreased the proliferative (Figure 4A, *P* < 0.05) and colony-forming (Figure 4B, *P* < 0.05) abilities of H460 and A549 cells. Furthermore, transfection with agomir-532-3p markedly increased the apoptotic rate of H460 and A549 cells (Figure 4C, *P* < 0.05). In addition, the results of the Transwell migration and invasiveness assays indicated that overexpression of miR-532-3p significantly attenuated the migration (Figure 4D, *P* < 0.05) and invasiveness (Figure 4E, *P* < 0.05) of H460 and A549 cells.

**Figure 4:** **miR-532-3p directly targets *HMGA2* mRNA to inhibit the malignant phenotype of NSCLC cells.** (**A**–**C**) Cell proliferation, colony formation, and apoptosis parameters determined by the CCK-8 assay, the colony formation assay, and flow cytometry in H460 and A549 cells transfected with agomir-532-3p or agomir-NC. *P < 0.05 vs. the agomir-NC group. (**D**, **E**) Migratory and invasive capabilities of H460 and A549 cells after transfection with agomir-532-3p or agomir-NC analyzed by the Transwell migration and invasiveness assays. *P < 0.05 vs. the agomir-NC group. (**F**) Wild-type and mutant miR-532-3p-binding site in the 3′-UTR of *HMGA2* mRNA. (**G**) Relative firefly luciferase activity determined in H460 and A549 cells at 48 h after co-transfection with agomir-532-3p or agomir-NC and *HMGA2*-wt or *HMGA2*-mut. *P < 0.05 vs. the agomir-NC group. (**H**) RT-qPCR analysis of *HMGA2* mRNA expression level in 51 pairs of NSCLC samples and corresponding normal lung tissues. *P < 0.05 vs. normal lung tissue. (**I**) Negative correlation between *HMGA2* mRNA and miR-532-3p levels in NSCLC tissue samples revealed by the Spearman’s correlation analysis (R^2^ = 0.3659, *P* < 0.0001). (**J, K**) *HMGA2* gene and protein expression levels in H460 and A549 cells determined by RT-qPCR and western blot, respectively, following transfection with agomir-532-3p or agomir-NC. *P < 0.05 vs. the agomir-NC group.

To uncover the molecular events underpinning miR-532-3p-mediated inhibition of NSCLC progression, the putative targets of this miRNA were searched in two bioinformatics databases. The bioinformatics prediction indicated that a site in the 3′-UTR of *HMGA2* mRNA matched the “seed sequence” of miR-532-3p (Figure 4F). HMGA2 was selected for further verification because that this gene was reported to be overexpressed in NSCLC and exert crucial roles during NSCLC initation and progression [29–32]. A luciferase reporter assay was then performed to demonstrate the possibility of miR-532-3p binding to the 3′-UTR of *HMGA2* mRNA in NSCLC cells. The luciferase activity of the HMGA2-wt reporter plasmid, which contained a wild-type miR-532-3p-binding site in the *HMGA2* 3′-UTR driving the expression of the luciferase gene, was notably weakened upon co-transfection of H460 and A549 cells with agomir-532-3p (*P* < 0.05). In contrast, the luciferase activity of HMGA2-mut was not altered by miR-532-3p upregulation (Figure 4G). In addition, RT-qPCR analysis confirmed that the mRNA expression of *HMGA2* was higher in the NSCLC tissue samples (Figure 4H, *P* < 0.05), revealing its negative correlation with the miR-532-3p expression level (Figure 4I; R^2^ = 0.3659, *P* < 0.0001). Moreover, transfection with agomir-532-3p significantly downregulated the mRNA (Figure 4J, *P* < 0.05) and protein (Figure 4K, *P* < 0.05) expression of *HMGA2* in H460 and A549 cells. Collectively, these data implied that miR-532-3p suppresses NSCLC progression and that *HMGA2* is a direct target gene of miR-532-3p.

### *VPS9D1-AS1* positively regulates *HMGA2* expression in NSCLC via sponging of miR-532-3p

As we established that *HMGA2* was a direct target gene of miR-532-3p in NSCLC cells, we next explored whether *VPS9D1-AS1* could modulate *HMGA2* expression in NSCLC cells. mRNA (Figure 5A, *P* < 0.05) and protein (Figure 5B, *P* < 0.05) levels of *HMGA2* were low in H460 and A549 cells deficient in *VPS9D1-AS1*, as revealed by RT-qPCR and western blot, respectively. To investigate whether miR-532-3p sponging mediated the positive effect of *VPS9D1-AS1* on *HMGA2* expression, rescue experiments were conducted in H460 and A549 cells by co-transfecting them with *si-VPS9D1-AS1* and antagomir-532-3p (inhibitor of miR-532-3p) or antagomir-NC. Transfection with antagomir-532-3p potently silenced miR-532-3p expression in H460 and A549 cells, as evidenced by RT-qPCR data (Figure 5C, *P* < 0.05). *VPS9D1-AS1* knockdown significantly increased miR-532-3p expression and decreased *HMGA2* mRNA and protein levels in H460 and A549 cells. In contrast, co-transfection with antagomir-532-3p abrogated the influence of *VPS9D1-AS1* knockdown on miR-532-3p (Figure 5D, *P* < 0.05) as well as on *HMGA2* mRNA (Figure 5E, *P* < 0.05) and protein (Figure 5F, *P* < 0.05) expression levels. These findings indicated that *VPS9D1-AS1* sponges miR-532-3p in NSCLC cells, thereby enhancing *HMGA2* expression.

**Figure 5:** ***VPS9D1-AS1* acts as a ceRNA of miR-532-3p and thereby upregulates *HMGA2* expression.** (**A**, **B**) *HMGA2* mRNA and protein levels in H460 and A549 cells determined by RT-qPCR and western blot, respectively, after transfection with *si-VPS9D1-AS1* or si-NC. *P < 0.05 vs. the si-NC group. (**C**) Efficiency of transfection of H460 and A549 cells with antagomir-532-3p determined by RT-qPCR. *P < 0.05 vs. the antagomir-NC group. (**D**–**F**) Expression levels of miR-532-3p, *HMGA2* mRNA, and HMGA2 protein in H460 and A549 cells after co-transfection with *si-VPS9D1-AS1* and antagomir-532-3p or antagomir-NC determined using RT-qPCR and western blot, respectively. *P < 0.05 vs. the si-NC group. ^#^*P* < 0.05 vs. the *si-VPS9D1-AS1* + antagomir-NC group.

### *VPS9D1-AS1* knockdown inhibits the malignant characteristics of NSCLC cells by reducing the miR-532-3p-*HMGA2* axis output

We carried out rescue experiments to further confirm that *VPS9D1-AS1* exerts its oncogenic effects in NSCLC cells by regulating the miR-532-3p-*HMGA2* axis. For this purpose, *si-VPS9D1-AS1* was co-transfected into H460 and A549 cells with antagomir-532-3p or antagomir-NC. As revealed by the CCK-8 assay, the colony formation assay, and flow cytometry, co-transfection with antagomir-532-3p reversed the modulatory influence of *VPS9D1-AS1* knockdown on the proliferation (Figure 6A, *P* < 0.05), colony-forming capacity (Figure 6B, *P* < 0.05), and apoptosis (Figure 6C, *P* < 0.05) of H460 and A549 cells, respectively. In addition, the suppression of H460 and A549 cell migration (Figure 6D, *P* < 0.05) and invasiveness (Figure 6E, *P* < 0.05) induced by *VPS9D1-AS1* knockdown was strongly attenuated by miR-532-3p inhibition.

**Figure 6:** **Inhibition of miR-532-3p strongly attenuates the influence of *VPS9D1-AS1* knockdown on the malignant characteristics of H460 and A549 cells.** (**A**–**E**) Proliferation, colony-forming capacity, apoptosis, migration, and invasiveness parameters of H460 and A549 cells measured by the CCK-8 assay, the colony formation assay, flow cytometry, Transwell migration and invasiveness assays, respectively. *P < 0.05 vs. the si-NC group. ^#^*P* < 0.05 vs. the *si-VPS9D1-AS1* + antagomir-NC group.

Rescue experiments were also performed in H460 and A549 cells after co-transfecting them with *si-VPS9D1-AS1* and the *HMGA2*-overexpressing plasmid pc-*HMGA2* or the corresponding empty pcDNA3.1 vector. Western blotting indicated that the downregulation of HMGA2 protein expression in *VPS9D1-AS1*-depleted H460 and A549 cells was almost completely reversed by the reintroduction of *HMGA2* (Figure 7A, *P* < 0.05). The CCK-8 and colony formation assays indicated that the restoration of *HMGA2* expression abrogated the inhibitory effects of *VPS9D1-AS1* knockdown on H460 and A549 cell proliferation (Figure 7B, *P* < 0.05) and colony formation (Figure 7C, *P* < 0.05). Similarly, the potentiation of H460 and A549 cell apoptosis by *VPS9D1-AS1* knockdown was prevented by co-transfection with pc-*HMGA2* (Figure 7D, *P* < 0.05). Transwell migration and invasiveness assays indicated that the restoration of *HMGA2* expression reversed the *si-VPS9D1-AS1*-induced inhibition of migration (Figure 7E, *P* < 0.05) and invasiveness (Figure 7F, *P* < 0.05) of H460 and A549 cells. In summary, *VPS9D1-AS1* knockdown attenuated *HMGA2* expression by reducing the sponging of miR-532-3p and thereby decreased NSCLC malignancy.

**Figure 7:** **Recovery of *HMGA2* expression reverses inhibitory actions of *si-VPS9D1-AS1* on NSCLC cells.** (**A**) Quantification of HMGA2 protein expression in H460 and A549 cells transfected with plasmid pc-*HMGA2* or the empty pcDNA3.1 vector along with *si-VPS9D1-AS1* by western blot. *P < 0.05 vs. the si-NC group. ^#^*P* < 0.05 vs. the *si-VPS9D1-AS1* + pcDNA3.1 group. (**B**–**F**) Cell proliferation, colony formation, apoptosis, migration, and invasiveness parameters of H460 and A549 cells, treated as described above, determined by the CCK-8 assay, the colony formation assay, flow cytometry, and Transwell migration and invasiveness assays, respectively. *P < 0.05 vs. the si-NC group. ^#^*P* < 0.05 vs. the *si-VPS9D1-AS1* + pcDNA3.1 group.

### *VPS9D1-AS1* knockdown slows down tumor growth of NSCLC cells *in vivo* by increasing miR-532-3p expression and decreasing *HMGA2* expression

We finally investigated the impact of *VPS9D1-AS1* knockdown on tumor growth *in vivo* in the xenograft experiment. H460 cells transfected with *si-VPS9D1-AS1* or si-NC were subcutaneously injected into nude mice. Tumor xenograft volume was much smaller in the *si-VPS9D1-AS1* group than in the si-NC group (Figure 8A, 8B; *P* < 0.05). In addition, tumor weight was significantly lower in the *si-VPS9D1-AS1* group than in the si-NC group (Figure 8C, *P* < 0.05) at 4 weeks after the injection of cells. *VPS9D1-AS1* expression was significantly downregulated in tumor xenografts from the si-VPS9D1-AS1 group, compared with that in xenografts from the si-NC group (Figure 8D, *P* < 0.05). Meanwhile, RT-qPCR revealed that miR-532-3p expression was higher in tumor xenografts derived from H460 cells transfected with si-VPS9D1-AS1 cells (Figure 8E, *P* < 0.05). Furthermore, HMGA2 protein expression was significantly lower in *the si-VPS9D1-AS1* group relative to that in the si-NC group (Figure 8F, *P* < 0.05). These results indicated that *VPS9D1-AS1* knockdown attenuated tumor growth of NSCLC cells through the downregulation of the miR-532-3p-HMGA2 axis output.

**Figure 8:** ***VPS9D1-AS1* knockdown suppresses tumor growth of NSCLC cells *in vivo*.** (**A**) Nude mice were inoculated with H460 cells transfected with *si-VPS9D1-AS1* or si-NC. Tumor volumes were measured 4 weeks after the injection, and tumor growth curves were plotted. *P < 0.05 vs. the si-NC group. (**B**) Representative images of tumor xenografts in the two groups. (**C**) Weights of tumor xenografts collected at the end of the experiment. *P < 0.05 vs. the si-NC group. (**D**, **E**) RT-qPCR analysis of *VPS9D1-AS1* and miR-532-3p expression levels in tumor xenografts from si-VPS9D1-AS1 and si-NC groups. *P < 0.05 vs. the si-NC group. (**F**) Western blot data illustrating the HMGA2 protein expression level in the tumor xenografts derived from H460 cells transfected with *si-VPS9D1-AS1* or si-NC. *P < 0.05 vs. the si-NC group.

## DISCUSSION

The differential expression of numerous lncRNAs in NSCLC has been extensively documented [33–35]. Changes in lncRNA expression levels affect a variety of pathophysiological characteristics associated with NSCLC [36–38]. Hence, the identification and characterization of lncRNAs aberrantly expressed in NSCLC will be useful for the development of new potential therapies for this deadly cancer. In this study, we quantitated *VPS9D1-AS1* expression in NSCLC tumors and cell lines. In addition, we examined the clinical value of monitoring the expression level of *VPS9D1-AS1* in patients with NSCLC. Furthermore, we investigated the regulatory functions of *VPS9D1-AS1* in NSCLC and revealed their molecular underpinnings. Collectively, the findings of our study provide insights for clinicians into the possible utility of targeting *VPS9D1-AS1* via the miR-532-3p-*HMGA2* axis for the management of NSCLC.

*VPS9D1-AS1* expression negatively correlates with tumor size and TNM stage in patients with gastric cancer [23]. Furthermore, patients with gastric cancer featuring low *VPS9D1-AS1* expression are expected to show shorter overall survival and shorter disease-free survival than patients with high *VPS9D1-AS1* expression [23]. In contrast, *VPS9D1-AS1* is overexpressed in prostate [24] and colorectal [25] cancers. These conflicting observations prompted our interest in establishing the expression profile of *VPS9D1-AS1* in NSCLC. We demonstrated that *VPS9D1-AS1* was upregulated in NSCLC tissue samples and NSCLC cell lines, in agreement with findings of another study [26]. In addition, we observed that the *VPS9D1-AS1* expression level was directly correlated with tumor size, TNM stage, and lymph node metastasis. Patients with NSCLC in the *VPS9D1-AS1* high-expression group exhibited shorter overall survival than patients in the *VPS9D1-AS1* low-expression group. These results suggest that *VPS9D1-AS1* might be a potential diagnostic and prognostic biomarker of NSCLC.

*VPS9D1-AS1* overexpression facilitates prostate cancer cell proliferation, colony formation, and migration [24]. We therefore sought to determine whether the aberrant upregulation of *VPS9D1-AS1* in NSCLC affected NSCLC malignancy. Several functional assays showed that *VPS9D1-AS1* knockdown by its siRNA attenuated NSCLC cell proliferation, migration, and invasiveness *in vitro*; moreover, it promoted apoptosis and attenuated tumor growth *in vivo*. These results implied that *VPS9D1-AS1* may be an effective target for NSCLC treatment.

Recently, lncRNAs have been proposed to function as “sponges” or “ceRNAs” in the regulatory network involving lncRNAs, miRNAs, and target genes [39–41]. In particular, *VPS9D1-AS1* has been demonstrated to work as a ceRNA of miR-184 and promote c-Myc expression in prostate cancer [24]. In the present study, we demonstrated that *VPS9D1-AS1* positively regulates *HMGA2* expression by acting as a ceRNA of miR-532-3p, thereby influencing NSCLC progression. First, we showed that *VPS9D1-AS1* mainly localizes in the cytoplasm of NSCLC cells, which supports the notion about its ceRNA properties. Secondly, *VPS9D1-AS1* was found to contain a complementary binding site for miR-532-3p; the binding and interaction between miR-532-3p and *VPS9D1-AS1* were verified in luciferase reporter and RIP assays. Thirdly, miR-532-3p expression was lower in NSCLC tissue samples and inversely correlated with *VPS9D1-AS1* expression. Fourthly, *VPS9D1-AS1* knockdown increased miR-532-3p levels but decreased *HMGA2* expression in NSCLC cells; these regulatory actions were reversed by miR-532-3p inhibition. Finally, the effects of *VPS9D1-AS1* knockdown on the malignant characteristics of NSCLC cells were neutralized by means of miR-532-3p inhibition or *HMGA2* reintroduction.

MiR-532-3p is downregulated in colorectal cancer [42], tongue squamous cell carcinoma [43], and ovarian cancer [44] but upregulated in hepatocellular carcinoma [45]. Expression of miR-532-3p is also low in NSCLC [46]. Nonetheless, the expression profile and functions of miR-532-3p in NSCLC have remained unclear. In this study, for the first time, we report that the aggressive phenotype of NSCLC is weakened by the upregulation of miR-532-3p, which directly targets *HMGA2* mRNA.

*HMGA2*, a member of the forkhead box transcription factor gene family [47], exerts important regulatory actions in chromatin architecture, gene transcription and replication by orchestrating the assembly of nucleoprotein complexes through a complex network of protein-DNA and protein-protein interactions [48, 49]; hence, *HMGA2* is implicated in the tumorigenesis and tumor development. *HMGA2* is highly expressed in NSCLC; its level correlates significantly with lymph node metastasis [29]. In addition, *HMGA2* level is an independent biomarker of NSCLC prognosis [29]. Functionally, *HMGA2* has been confirmed as an oncogene during NSCLC initiation and progression [30–32]. Here, we proved that *HMGA2* expression is positively regulated by *VPS9D1-AS1* in NSCLC; further, we showed that this regulatory effect is essential for the tumorigenic actions of *VPS9D1-AS1* in NSCLC cells. *VPS9D1-AS1* acts as a sponge on miR-532-3p to restrict its suppressive effect on *HMGA2* expression, thus augmenting the aggressive phenotype of NSCLC cells *in vitro* and *in vivo*. Apparently, the *VPS9D1-AS1*-miR-532-3p-*HMGA2* pathway is important for the malignant manifestations of NSCLC, which makes it an attractive target for NSCLC therapy.

There are three limiations in our current study. First, we detected VPS9D1-AS1 expression in only 51 paired samples of NSCLC and corresponding normal lung tissues. In our following experiments, we will collect more tissue specimens and further validate our finding. Second, HMGA2 was identified as a direct target gene of miR-532-3p. However, further studies are still necessary to explore whether there are other targets of miR-532-3p and examine whether they could play a role in NSCLC tumorigenesis. Finally, NSCLC is comprised mainly of three subtypes, which are widely accepted to be different diseases. Nevertheless, we did not examine the correlation between VPS9D1-AS1 expression and NSCLC subtypes. We will resolve these limitations in the near future.

## CONCLUSION

This study provides important insights into the expression profile and tumorigenic properties of *VPS9D1-AS1* lncRNA in NSCLC malignancy. The oncogenic effects of *VPS9D1-AS1* in NSCLC are likely mediated via its sponging of miR-532-3p and the consequent increase in *HMGA2* expression. The components of the regulatory pathway that includes *VPS9D1-AS1*, miR-532-3p, and *HMGA2* may serve as potential targets for novel therapeutic approaches to treat NSCLC.

## MATERIALS AND METHODS

### Ethics statement

This study was conducted in accordance with the ethical standards recommended by the Declaration of Helsinki and according to national and international guidelines. The study was approved by the institutional review boards of the authors' institutions. In particular, the experimental procedures of this study were approved by the Ethics Committee of the Cancer Hospital of the Guangxi Medical University. Written informed consent was also obtained from all patients before their enrolment in this study. The experimental procedures involving animals were approved by the Animal Ethics Committee of the Cancer Hospital of the Guangxi Medical University, and the assays were carried out in accordance with the Animal Protection Law of the People’s Republic of China-2009 for experimental animals.

### Clinical tissue specimens

Paired samples of NSCLC and corresponding normal lung tissues were obtained from 51 patients with NSCLC who underwent surgical resection at the Cancer Hospital of the Guangxi Medical University. None of the patients were treated with chemotherapy, radiotherapy, or other anticancer modalities prior to the surgical intervention. All tissue specimens were immediately frozen in liquid nitrogen and preserved at −80°C until further use.

### Cell culture

Normal non-tumorigenic bronchial epithelium cell line BEAS-2B and five human NSCLC cell lines (H522, H460, H1299, A549, and SK-MES-1) were purchased from the Cell Bank of the Type Culture Collection of the Chinese Academy of Sciences (Shanghai, China). Dulbecco’s modified Eagle’s medium (DMEM) containing 10% fetal bovine serum (FBS) and 1% (v/v) of a penicillin-streptomycin solution (Gibco; Thermo Fisher Scientific, Inc., Waltham, MA, USA) was utilized for cell culture. All cells were maintained in a humidified atmosphere of 95% air and 5% CO_2_ at 37°C.

### Transfection procedures

The siRNA that specifically reduced the expression of *VPS9D1-AS1* (si-VPS9D1-AS1) and si-NC were acquired from RiboBio Biotechnology (Guangzhou, China). miR-532-3p agomir (agomir-532-3p), negative control agomir (agomir-NC), antagomir-532-3p, and antagomir-NC were designed and chemically produced by GenePharma (Shanghai, China). The constructed *HMGA2* overexpression plasmid pcDNA3.1-*HMGA2* (pc-*HMGA2*) and the empty pcDNA3.1 vector were purchased from IBSbio (Shanghai, China). The cells were seeded into 6-well plates, and all transfection procedures were conducted using the transfection reagent Lipofectamine 2000 (Invitrogen; Thermo Fisher Scientific, Inc.).

### Subcellular fractionation and RT-qPCR

The cytoplasmic and nuclear fractions of NSCLC cells were separated using a PARIS kit (Ambion; Thermo Fisher Scientific, Inc.). RNA was isolated from both fractions and analyzed by RT-qPCR.

Total RNA was isolated using TRIzol® reagent (Invitrogen; Thermo Fisher Scientific, Inc., USA) and quantified on a NanoDrop 2000c spectrophotometer (Invitrogen; Thermo Fisher Scientific, Inc.). An All-in-One™ miRNA qRT-PCR Detection Kit (GeneCopoeia, Rockville, Md, USA) was used to determine the miR-532-3p expression, with *U6* small nuclear RNA as control. *HMGA2* mRNA and *VPS9D1-AS1* expression levels were measured using a PrimeScript RT Reagent Kit and SYBR Premix Ex Taq™ (Takara Biotechnology Co., Ltd., Japan). The *GAPDH* mRNA level served as the internal reference for *HMGA2* mRNA and *VPS9D1-AS1* expression levels. The relative gene expression level was calculated by the 2^−ΔΔCq^ method [50].

### CCK-8 assay

Transfected cells were detached using 0.25% trypsin, counted, and seeded into 96-well plates at a density of 2 × 10^3^ cells/well. The cells were maintained at 37°C and 95% O_2_/5% CO_2_. The medium in each well was supplemented with 10 μL of the CCK-8 solution (Dojindo Molecular Technologies, Inc., Kumamoto, Japan) at 0, 24, 48, and 72 h post seeding. Cell proliferation rate was inferred from the optical density values at 450 nm measured on a microplate reader (Molecular Devices, Sunnyvale, CA, USA).

### Colony formation assay

In total, 2 mL of a cell suspension containing 1,000 transfected cells was seeded into each well of 6-well plates. After 2 weeks of incubation in a humidified atmosphere of 95% air and 5% CO_2_ at 37°C, the cells were fixed in 100% methanol, stained with methyl violet (Beyotime Institute of Biotechnology, Inc., Shanghai, China), and extensively washed with phosphate buffered saline (Gibco; Thermo Fisher Scientific, Inc.). The number of colonies (≥50 cells) was determined under an inverted microscope (Olympus, Tokyo, Japan).

### Flow cytometry

After 48 h of culture, transfected cells were harvested with 0.25% trypsin without EDTA, washed thrice with phosphate buffered saline, and centrifuged. An Annexin V-Fluorescein Isothiocyanate (FITC) Apoptosis Detection Kit (Biolegend, San Diego, CA, USA) was employed to determine cell apoptosis rates. Cells were resuspended in 100 μL of binding buffer and stained with 5 μL of Annexin V-FITC and 5 μL of propidium iodide solution. Following a 15 min incubation in the dark at room temperature, the apoptotic cells were scored using a FACScan flow cytometer (BD Biosciences, CA, USA).

### Transwell migration and invasiveness assays

Matrigel (BD Biosciences) diluted with DMEM was utilized to coat the Transwell chambers (BD Biosciences) for the Transwell invasiveness assay but not for the migration assay. Transfected cells were harvested at 48 h post-transfection, washed twice with phosphate-buffered saline, and resuspended in FBS-free DMEM. In total, 50,000 cells were plated into the upper compartments and 500 μL of DMEM supplemented with 20% FBS was added into the lower compartments. Later, the chambers were placed into a 37°C incubator supplied with 95% air/5% CO_2_ for 24 h incubation; then, the cells remaining on the inner side of the membranes were wiped off with cotton balls. Migratory and invasive cells were fixed with 100% methanol and stained with 0.1% crystal violet. After extensive washing, migratory and invasive cells were photographed under an inverted microscope. Five fields of view were randomly selected, and the average numbers of migratory and invasive cells were determined.

### Tumor xenograft experiment

Four-week-old nude mice were bought from the Guangdong Medical Laboratory Animal Center (Foshan, Guangdong, China) and randomly divided into two groups. One group was subcutaneously injected with *si-VPS9D1-AS1*-transfected H460 cells, whereas the other group was similarly injected with si-NC-transfected H460 cells. The volume of tumor xenografts was calculated according to the following formula: volume (mm^3^) = (L × W^2^)/2; where L and W represent the length (longest dimension) and width (shortest dimension), respectively. At the end of the experiment, all mice were euthanized, and tumor xenografts were collected for further analysis.

### RIP assay

The RIP assay was conducted using a Magna RIP RNA-Binding Protein Immunoprecipitation Kit (Millipore Inc., Billerica, MA, USA). In brief, cells were lysed with RIPA lysis buffer and centrifuged at 14,000 rpm for 10 min at 4°C. The supernatant was incubated with magnetic beads conjugated with anti-Argonaute 2 (AGO2) or anti-IgG antibodies (Millipore Inc.). After overnight incubation at 4°C, the immunoprecipitated RNA was purified using proteinase K digestion and analyzed by RT-qPCR.

### Bioinformatics prediction

We searched for miRNA(s) that could be sponged by *VPS9D1-AS1* using starBase 3.0 (http://starbase.sysu.edu.cn/). The putative targets of miR-532-3p were predicted using two publicly available databases: miRDB (http://mirdb.org/) and TargetScan (http://www.targetscan.org/vert_60/).

### Luciferase reporter assay

The fragments of *VPS9D1-AS1* containing wt or mut miR-532-3p binding site were PCR-amplified by GenePharma and inserted into the pmirGLO luciferase reporter vector (Promega Corporation, Madison, WI, USA) to create recombinant reporter plasmids VPS9D1-AS1-wt and VPS9D1-AS1-mut. The construction of luciferase reporter plasmids *HMGA2*-wt and *HMGA2*-mut was performed in a similar manner.

H460 and A549 cells were seeded in 24-well plates one night before the transfection. Wt or mut recombinant plasmids and agomir-532-3p or agomir-NC were co-transfected into NSCLC cells using Lipofectamine 2000. At 48 h post-transfection, the cells were collected and subjected to the Dual-Luciferase Reporter Assay (Promega Corporation) to measure the firefly and *Renilla* luciferase activities. The activity of the firefly luciferase was normalized to that of the *Renilla* luciferase.

### Western blot analysis

Total protein was extracted using RIPA lysis buffer and quantified using the BCA Protein Assay Kit (Beyotime, Shanghai, China). Equal amounts of proteins were separated by sodium dodecyl sulfate 10% polyacrylamide gel electrophoresis and transferred onto polyvinylidene difluoride membranes. Unoccupied sites on the membranes were blocked with 5% nonfat milk diluted with Tris-buffered saline containing 0.1% Tween 20 (TBST) for 2 h at room temperature. After incubation with primary antibodies against HMGA2 (ab207301; dilution 1:1,000) or GAPDH (ab181602; dilution 1: 1,000; both from Abcam, Cambridge, UK) overnight at 4°C, the membranes were extensively washed with TBST and incubated with a goat anti-rabbit IgG antibodies conjugated with horseradish peroxidase (ab205718; dilution 1:5,000; Abcam, Cambridge, UK). After three washes, the signals were detected using an Enhanced Chemiluminescence Western Blotting Detection Kit (Applygen Technologies, Inc., Beijing, China).

### Statistical analysis

All data were analyzed using SPSS statistical software (version 11.0; SPSS, Inc.) and are presented as the mean ± standard deviation. Pairwise comparisons were performed using Student’s *t* test, whereas statistical analysis of multiple groups (≥3) was carried out using one-way analysis of variance, followed by the post hoc Tukey’s test, if appropriate. The correlation between *VPS9D1-AS1* and miR-532-3p expression levels in NSCLC tissue samples was established using the Spearman’s rank correlation analysis. The association between *VPS9D1-AS1* level and the clinicopathological characteristics of patients with NSCLC was examined using the chi-squared test. The overall survival rates of NSCLC patients were analyzed by the Kaplan–Meier method and compared by the log-rank test. All statistical analyses were conducted at a significance level of α = 0.05 (*P* < 0.05).
